# Modulation of Sustained Attention by Theta-tACS over the Lateral and Medial Frontal Cortices

**DOI:** 10.1155/2021/5573471

**Published:** 2021-06-19

**Authors:** Jinwen Wei, Zhiguo Zhang, Ziqing Yao, Dong Ming, Peng Zhou

**Affiliations:** ^1^School of Precision Instrument and Optoelectronics Engineering, Tianjin University, Tianjin 300072, China; ^2^School of Biomedical Engineering, Health Science Center, Shenzhen University, Shenzhen 518060, China; ^3^Department of Psychology, The University of Hong Kong, Hong Kong S.A.R., China

## Abstract

Theta oscillations over the posterior medial frontal cortex (pMFC) and lateral prefrontal cortex (LPFC) play vital roles in sustained attention. Specifically, pMFC power and pMFC-LPFC synchronization correlate with cognitive control in sustained-attention-related tasks, but the causal relationships remain unknown. In the present study, we first analyzed the correlation between EEG theta oscillations (characterized by time-frequency power and phase-based connectivity) and the level of sustained attention (Experiment 1) and then utilized transcranial alternating current stimulation (tACS) to modulate theta oscillations and in turn observed its effects on sustained attention (Experiment 2). In Experiment 1, two time-frequency regions of interest (ROIs) were determined, in which high/low time-frequency power and high/low phase-based connectivity corresponded to high/low-level sustained attention. In Experiment 2, time-frequency power and phase-based connectivity of theta oscillations were compared between the sham and tACS groups within the time-frequency ROIs determined in Experiment 1. Results showed that phase-based connectivity between pMFC and LPFC significantly decreased in the tACS group compared with the sham group during the first five minutes of the poststimulation period. Moreover, a marginal trend existed that sustained attention was downregulated by tACS in the same time interval, suggesting that theta phase synchronization between pMFC and LPFC may play a causal role in sustained attention.

## 1. Introduction

Sustained attention could be defined as “the ability to self-sustain mindful, conscious processing of stimuli whose repetitive, non-arousing qualities would otherwise lead to habituation and distraction to other stimuli” [1]. Although debates still exist about how sustained attention fits into the overall taxonomy of attention or cognition [2], it is widely accepted that sustained attention constitutes key parts of attention, especially alerting and orienting networks [3, 4]. Sustained attention is also very sensitive to disorders and damage of the brain, such as traumatic brain injury [1] and attention-deficit hyperactivity disorder [5]. Therefore, it is of great significance to pinpoint the neural mechanisms of sustained attention.

A large number of studies have suggested that sustained attention correlates closely with cortical oscillations, extracted often from electroencephalography (EEG) signals. Integrated into the model proposed by Clayton et al., frontomedial theta (fm-theta) oscillations and the coordination between the posterior medial frontal cortex (pMFC) and the lateral prefrontal cortex (LPFC) play vital roles in sustained attention [6]. Specifically, fm-theta power relates to monitoring and control functions in attention-related tasks. For example, fm-theta power has been shown to significantly increase following the presentation of rare oddball stimuli and negative task feedback [7, 8]. On the other hand, theta phase synchronization allows theta-driven cognitive monitoring systems to exert control over attention via connecting the pMFC and LPFC [6]. For example, theta phase synchronization between pMFC and LPFC increased significantly during high response conflicts [9] or following negative feedback [8], both demanding an effective transmission of information between these two brain areas. However, regardless of fm-theta power, pMFC-LPFC theta phase synchronization, or other oscillatory features, whether they are merely correlated or have causal relationships with sustained attention remains unknown.

Transcranial alternating current stimulation (tACS), a noninvasive brain stimulation technique, is capable of providing causal evidence concerning the role of cortical oscillations in cognition [10, 11]. By using tACS to modulate a specific cortical oscillation and observing the physiological responses accompanied by behavioral consequences, we can infer the causal relationship between these cortical oscillations and cognitive functions. For example, frontotemporal theta tACS with an in-phase protocol significantly improved working memory by synchronizing cortical oscillations [12]. TACS has also been demonstrated to modulate sustained attention through stimulating pMFC [13, 14] or the occipitoparietal cortex [15, 16], yet their effects were inconsistent. Given that pMFC-LPFC synchronization plays a crucial role in sustained attention, we expected that applying tACS could modulate theta-band pMFC-LPFC oscillations and ultimately affect sustained attention.

The present study is aimed at investigating the causal roles of theta-band pMFC-LPFC oscillations in sustained attention via tACS. To this end, we conducted two close-knit experiments in two steps. In Experiment 1, we used EEG to explore whether and how theta-band pMFC-LPFC oscillations were correlated with sustained attention. Two types of EEG features—time-frequency power on pMFC and phase-based connectivity between pMFC and LPFC—were analyzed. Based on the correlative evidence between these two features and the sustained attention obtained from Experiment 1, we further conducted Experiment 2 by applying theta-tACS (6 Hz) to specifically modulate the power as well as phase synchronization between pMFC and LPFC to affect the behavioral performance of sustained attention. Experiment 2 was expected to provide causal evidence between theta-band pMFC-LPFC oscillations and sustained attention, which would be fundamentally helpful in advancing our understanding of the neural mechanisms of sustained attention.

## 2. Materials and Methods

### 2.1. Experiment 1

#### 2.1.1. Participants

A total of 10 volunteers (6 males, mean age 22.2 ± 1.5 years) participated in this study. All participants were on-campus students and had a normal or corrected-to-normal vision. None of them suffered from any neurological or psychological disorder or took medication that interfered with the study. Before formal participation, they were required to rest well and to refrain from consuming caffeine or alcohol. Participants provided informed consent before the start of the experiment. The experiment was approved by the local ethics committee at Tianjin University.

#### 2.1.2. Task

The psychomotor vigilance task (PVT) is a simple but mentally demanding reaction time test, which is often used in research on sustained attention and fatigue [17]. In the present study, a 30 min version of PVT was administered (Figure 1). During the test, subjects were required to monitor three adjacent boxes representing a millisecond counter. Once the counter occurred in the center of a computer monitor, they needed to respond by pressing the space bar as quickly as possible. Subjects were given a maximum of 1 s to stop the counter and received their reaction time (RT) after the counter was presented. The interval of counters was 2-10 s (mean = 6 s), and the task included 300 trials in total. The stimulus presentation was programmed with the Psychophysics Toolbox Version 3 (http://psychtoolbox.org) for MATLAB (The MathWorks, Inc., Natick, MA, US).

#### 2.1.3. EEG Recording and Processing

EEG signals were acquired from 64 Ag/AgCl scalp electrodes at 1000 Hz using the Neuroscan EEG acquisition apparatus (Neuroscan Inc., USA) according to the international 10-20 system. Electrode impedances were kept below 10 k*Ω* during the whole experiment. After recording, raw EEG signals were cleaned from clear artifacts by visual inspection, filtered by high-pass filter with 0.1 Hz using EEGLAB software [18], and rereferenced offline to the average of both left and right mastoid sites. Then, the independent component analysis (ICA) was done to separate eye movements, eye blinks, and other noise artifacts. The independent components were visually inspected, and those representing artifacts were removed.

### 2.2. Behavioral Analysis

The RTs of the trials were computed in custom-written MATLAB programs. Firstly, to see the overall trend of sustained attention, we presented RTs averaged across all subjects. Secondly, all trials were rearranged sequentially from short to long RT. Then, the first one-third trials were grouped and analyzed as representing high-level sustained attention, and the last one-third trials were grouped and analyzed as low-level sustained attention, as similarly done in the previous study [19]. Subsequently, a paired *t*-test with average reaction time as dependent variables in two trial groups (i.e., the high- and low-level sustained attention) was run to determine if there were differences between high-level and low-level sustained attention. Trials with longer than 500 ms and shorter than 200 ms (approximately 10%) were excluded from the analysis. To justify the sample size involved in Experiment 1, we reported Cohen's *d* effect sizes where an effect size of 0.2 is small, 0.5 is medium, 0.8 is large, and 1.2 is very large [20]. Also, we conducted Bayesian analysis and report Bayes factor (BF), which is essentially the ratio between the odds of the posterior (observed) model and the odds of the null model. Typically, a factor of 3–10 is considered “moderate” evidence, a factor of 10–30 is considered “strong” evidence, and a factor of larger than 30 is considered to be “very strong” evidence against the null model [21].

### 2.3. EEG Oscillation Analysis

#### 2.3.1. Time-Frequency Power

First, EEG data were segmented into epochs from -1000 ms to 1200 ms relative to the onset of the stimulus. According to RTs, the epochs corresponding to two levels of sustained attention, the same way as behavioral analysis did, were selected. Next, single-trial epochs were decomposed into their time-frequency representation via convolution with a family of complex Morlex wavelets, defined as Gaussian-tapered complex sine waves. Forty logarithmically spaced frequencies between 2 Hz and 40 Hz were utilized. The number of cycles increased from 3 to 10 in logarithmical steps. The convolution was conducted through frequency-domain multiplication, in which the Fourier-derived spectrum of epochs was multiplied by the spectrum of wavelets, and then, the inverse Fourier transform was performed. Power and phase were defined and thus extracted as the squared magnitude of the complex result and the angle relative to the positive real axis, respectively. Note that the power was normalized using a decibel (dB) transform (dB power = 10∗log10 [power/baseline]), where the baseline was the average power at each frequency band from −400 ms to −200 ms before the onset of the stimulus and the time range from -200 ms to 800 ms was presented. To find significant different regions in the whole time-frequency domain, a cluster-based permutation test was used [22]. Power data under two conditions (high- and low-level sustained attention) were shuffled in each subject 1000 times. The random data were then used to establish null distributions of effects under the existing bias. Next, clusters of temporally and spectrally adjacent significant differences (threshold *p* < 0.05) were identified. The sum of *t* values in each cluster was calculated in the original data and the permutated data. If no *t* value reached significance in one of the permutations, a cluster value of 0 was assigned. The significance of clusters was assessed by calculating the rank of the cluster *t* values in the distribution of random data. A cluster was interpreted as significant if an absolutely higher cluster *t* -value was found in less than 5% of the random permutations. Finally, the time-frequency regions of interest (ROIs) for power analysis were determined based on those significant clusters, and a paired *t*-test was utilized to compare the averaged power within that determined window between high-level and low-level sustained attention.

#### 2.3.2. Phase-Based Connectivity

Phase-based connectivity is also known as phase synchronization or phase coherence [23]. Here, we used the debiased weighted phase lag index (dWPLI) [24] to estimate phase-based connectivity. This index weights phase angle differences according to their distance from the real axis such that vectors closer to the real axis have a smaller influence on the estimation of connectivity. The dWPLI between two channels is calculated in

(1) $$\begin{array}{c} \text{dWPLI}=\frac{\sum_{j=1}^{N}\sum_{k\neq j}I\left\{X_{j}\right\}I\left\{X_{k}\right\}}{\sum_{j=1}^{N}\sum_{k\neq j}\left|I\left\{X_{j}\right\}I\left\{X_{k}\right\}\right|}, \end{array}$$

in which *N* is the number of trials and *ℑ*{} denotes the imaginary part of the cross-spectrum *X* between two electrodes. Compared with other indexes, such as phase-locking value (PLV), dWPLI is more insensitive to volume conduction and more appropriate for exploratory data-driven studies. Note that the spatial filter of the surface Laplacian [25], also known as “current source density” or “current scalp density”, was applied for all epochs before computing dWPLI. This procedure would substantially increase topographical selectivity and attenuate volume conduction, which has been demonstrated to be an important and necessary step to the electrode-level connectivity analysis [23, 26].

The Fz and F3 electrodes were used to measure activities over pMFC and LPFC, respectively, consistent with prior studies [27–30]. Then, the dWPLI between Fz and F3 was presented in the time-frequency domain under two levels of sustained attention. It should be noted that because the dWPLI here was necessarily calculated by averaging across trials, so it is not feasible to compute cluster-based permutation to find significant difference areas. Instead, we selected an interested time-frequency window via visually choosing the difference map between high-level and low-level sustained attention. Then, a paired *t*-test was utilized to compare the averaged dWPLI within that selected window.

### 2.4. Experiment 2

#### 2.4.1. Participants

Fifteen volunteers (8 males, mean age 22.8 ± 1.2 years) who had a normal or corrected-to-normal vision and were also naïve concerning the stimulation participated in this study. Every participant took part in two experimental sessions: sham stimulation and tACS. The periods between the two sessions ranged from 1 day to 1 week. The sequence of applying two sessions was counterbalanced across subjects. All subjects provided informed consent before the start of the experiment. Influences of circadian rhythms were minimized by scheduling the sessions for all participants only in the afternoon. Three participants were excluded due to insufficient EEG data after preprocessing, leaving twelve participants (6 males) for analysis. The experiment was approved by the local ethics committee at Tianjin University.

#### 2.4.2. Task

In Experiment 2, we used a revised version of the psychomotor vigilance test (Figure 2). Participants needed to respond by pressing the space bar as quickly as possible once a red circle presented in the center of the monitor. Subjects were given a maximum of 1 s to react to the circle, and then, a smile or sad expression was presented as feedback. The type of expression depended on whether the reaction time exceeded the threshold. If the reaction time exceeded the threshold, there would be a sad expression and vice versa. During the first 5 minutes, the threshold of 350 ms (equals the average plus the standard deviation of the reaction time across participants in Experiment 1) was set. In the remaining 25 minutes, the threshold was the average plus the standard deviation of the reaction time in the first 5 minutes. This adaptive threshold was applied to involve participants' reactions based on different baseline states in the two stimulation groups. The interval of counters was 2-10 s (mean = 6 s), and the task contained 300 trials in total. The stimulus presentation was programmed with the Psychophysics Toolbox Version 3 (http://psychtoolbox.org) for MATLAB (The MathWorks, Inc., Natick, MA, US).

### 2.5. Transcranial Alternating Current Stimulation (tACS)

tACS was delivered by a battery-operated stimulator (DC-Stimulator Plus, neuroConn, Germany). The stimulator was connected to two Ag/AgCl electrodes with a 1 cm radius, which thus provided *π* circular area for each one. The electrodes named PISTIM, produced by Neuroelectrics, Spain, can work for both stimulation and EEG monitoring. Based on the fact that sustained attention was highly correlated with theta-band oscillations in Experiment 1, a sinusoidally alternating current of 1 mA (peak-to-peak) was applied at 6 Hz continuously lasting for 15 minutes. Six Hz was selected here as the center frequency in two interested frequency bands, 4-6 Hz and 5-8 Hz, obtained from Experiment 1. The stimulating current was ramped up over 20 seconds to 1 mA in both sham stimulation and tACS groups; however, the current was then faded into 0 mA in 20 seconds in the sham group. Participants reported that neither painful skin sensations nor phosphenes were induced, and particularly, they could not distinguish between the sham and tACS groups. Specifically, the phase difference between the two stimulating electrodes was set at 180° determined by the stimulation montage we used in this experiment.

### 2.6. Behavioral Analysis

For every participant under each stimulation (sham stimulation or tACS), the behavior baseline was defined by the sum of the mean and the standard deviation of reaction times in the first 5 minutes. To rule out the possible confounding effect of individual baseline differences, we chose not to compare RTs directly, but the proportions of negative responses as follows. First, we specified six time intervals, namely, 0-5 min, 5-10 min,…, 20-25 min, and 25-30 min, respectively. Next, within each time interval, the number of sad expressions was divided by the number of all expressions. Last, these ratios of sad expressions (i.e., proportions of negative responses) in six time intervals (within-subject factor, 6 levels) under two conditions (sham/tACS, within-subject factor, 2 levels) were compared using two-way repeated measures ANOVA. Furthermore, to investigate the immediate effects after stimulation, considering the nonuniformity of behavioral data in the current dataset, the Wilcoxon signed-rank test on paired samples was performed to compare sustained attention in the fifth time interval (20-25 min) between the sham and tACS groups. To justify the sample size involved in Experiment 2, we report effect size estimates used with the Wilcoxon signed-rank test where an effect size *r* of 0.10-0.30 is small, 0.30-0.50 is medium, and bigger than 0.50 is large [31]. Also, we conducted Bayesian rank-based hypothesis testing for the signed-rank test [32] and report Bayes factor (BF), which is essentially the ratio between the odds of the posterior (observed) model and the odds of the null model. Typically, a factor of 3–10 is considered “moderate” evidence, a factor of 10–30 is considered “strong” evidence, and a factor of larger than 30 is considered to be “very strong” evidence against the null model [21].

### 2.7. EEG Analysis

Because EEG signals during the stimulation (5-20 min) were introduced large amounts of artifacts, so we only analyzed the signals right before the stimulation (0-5 min) and right after the stimulation (20-30 min). Artifacts were cleaned by first visual inspection and then ICA. On average, 20% of the trials were rejected. As a consequence, for every participant, approximately 40 trials remained in the first 5 minutes, and approximately 80 trials remained in the last 10 minutes. We used those 40 trials in the first 5 minutes to represent the state of sustained attention before stimulation, and those 80 trials in the last 10 minutes to represent the state of sustained attention after stimulation.

The time-frequency decomposition is the same as that in Experiment 1. The interested time-frequency windows determined in Experiment 1 were utilized to examine the difference between the sham and tACS groups. Within those windows, the averaged time-frequency power change at electrode Fz and the averaged phase-based connectivity change at Fz-F3 in the last two time intervals (i.e., 20-25 min and 25-30 min, within-subject factor, 3 levels), relative to the baseline (0-5 min), under two stimulations (i.e., sham and true tACS, within-subject factor, 2 levels) were compared using two-way repeated measures ANOVA. The relative change was used here due to different baseline states [33]. Note that these time intervals do not have the same length; instead, the time interval of 0-5 min consists of all remaining trials in the first 5 minutes, and the second as well as the third time interval equally divided 1/2 of the remaining trials in the last 10 minutes. We argued that this implementation was feasible because the rejected trials (about 20%) were randomly distributed over time.

Furthermore, to investigate the immediate effects after stimulation, considering the nonuniformity of time-frequency data, the Wilcoxon signed-rank test on paired samples was performed to compare power and phase synchronization in the fifth time interval (20-25 min) between the sham and tACS groups, a similar way conducted in the previous tACS study [34].

## 3. Results

### 3.1. Experiment 1

#### 3.1.1. Behavioral Results

Figure 3 shows the behavioral data (RT) in Experiment 1. Averaged RTs increased with experimental time, indicating that the level of sustained attention gradually decreased (Figure 3(a)). Statistical results showed that the mean RT of high-level sustained attention trials (313.28 ± 21.96 ms) was significantly faster than that of low-level sustained attention trials (420.80 ± 25.92 ms), *t* (9) = −30.42, *p* < 0.0001, corresponding to Cohen's *d* effect size of *d* = 9.62 (a very large effect). These results indicated that high-level and low-level sustained attention can be well distinguished by their RTs in Experiment 1 (Figure 3(b)). A similar conclusion was also reached by Bayesian *t*-tests, which showed extremely strong evidence against the null hypothesis that there was no difference in RTs between high-level and low-level sustained attention (BF > 1000).

#### 3.1.2. EEG Time-Frequency Power

Time-frequency power on the pMFC (electrode Fz) was averaged across all subjects under high-level and low-level sustained attention, respectively (Figures 4(a) and 4(b)). Time-frequency points with significant differences between high-level and low-level sustained attention were revealed by the cluster-based permutation test and were indicated by thin lines in Figure 4(c). Based on the results shown in Figure 4(c) as well as the predetermined interest of the theta band, the interested time-frequency window was chosen to be 150-350 ms and 4-6 Hz, as indicated by the bold black rectangle in Figure 4(c). Within this time-frequency window, the averaged power of high-level sustained attention (1.46 ± 1.18 dB) was significantly larger than that of low-level sustained attention (−0.08 ± 1.32 dB) with *t* (9) = 3.30, *p* < 0.01 (Figure 4(d)), corresponding to Cohen's *d* effect size of *d* = 1.04 (a large effect). A similar conclusion was also reached by Bayesian *t*-tests, which showed moderate evidence against the null hypothesis that there was no power difference in the specified time-frequency window between high-level and low-level sustained attention (BF = 6.62).

#### 3.1.3. Phase-Based Connectivity

DWPLI between pMFC (Fz) and LPFC (F3) was averaged across all subjects under high-level and low-level sustained attention, respectively (Figures 5(a) and 5(b)).  Figure 5(c) shows the difference of dWPLI between high-level and low-level sustained attention (high-level minus low-level). The interested time-frequency window was visually selected to be 150-300 ms and 5-8 Hz, as indicated by the bold black rectangle in Figure 5(c). Within this time-frequency window, the averaged dWPLI of high-level sustained attention (0.11 ± 0.12) was significantly larger than that of low-level sustained attention (0.02 ± 0.05), with *t* (9) = 2.68, *p* < 0.05 (Figure 5(d)), corresponding to Cohen's *d* effect size of *d* = 0.846 (a large effect). A similar conclusion was reached by Bayesian *t*-tests, which showed nearly moderate evidence against the null hypothesis that there was no dWPLI difference in the specified time-frequency window between high-level and low-level sustained attention (BF = 2.97).

Taken together, two different time-frequency windows were specified in which high-level sustained attention had both larger power and larger phase-based connectivity than low-level sustained attention in Experiment 1.

### 3.2. Experiment 2

#### 3.2.1. Behavioral Results

A two-way repeated measures ANOVA was run to determine the effect of different stimulations (sham/tACS) over time intervals (0-5, 5-10,…, 25-30 min) on sustained attention, represented by the proportions of negative responses. The interaction effect between stimulation and time intervals on sustained attention was not statistically significant, *F* (5, 55) = 0.448, *p* = 0.81, partial *η*^2^ = 0.01. The main effect of stimulation was nonsignificant, *F* (1, 11) = 0.730, *p* = 0.411, partial *η*^2^ = 0.012. The main effect of time intervals yielded an *F* ratio of *F* (5, 55) = 12.402, *p* < 0.001, indicating that the levels of sustained attention varied significantly across time intervals and sustained attention declined with the experimental time going on (see Figure 6(a) and multiple comparisons for time intervals in Table 1). To specifically see the immediate effects just after different stimulations over the fifth time interval (the first time interval in the poststimulation period) on sustained attention, a left tailed Wilcoxon signed-rank test on paired samples was conducted and the results showed that the negative proportion change of the sham group has a nonsignificantly declining trend compared to that of the tACS group, *p* = 0.068, corresponding to an effect size *r* = 0.442 (a medium effect). These results indicated that tACS probably reduced sustained attention when the tACS was terminated (see Figure 6(b)). On the other hand, Bayesian analysis showed small evidence against the null hypothesis that sustained attention was up(non)-regulated in tACS condition (BF = 1.96).

#### 3.2.2. Time-Frequency Power

A two-way repeated measures ANOVA was run to determine the effect of different stimulations (sham/tACS) over time intervals (20-25 min and 25-30 min) on the averaged power change relative to baseline (0-5 min) within the time-frequency window (150-350 ms, 4-6 Hz) determined in Experiment 1 (Figure 6(c)). The interaction effect between stimulation and time interval on averaged power was not statistically significant, *F* (1, 11) = 0.005, *p* = 0.947, partial *η*^2^ = 0.00004. The main effect of stimulation was nonsignificant, *F* (1, 11) = 0.031, *p* = 0.864, partial *η*^2^ = 0.001. The main effect of time intervals was nonsignificant, *F* (1, 11) = 1.158, *p* = 0.305, partial *η*^2^ = 0.007. To specifically see the immediate effect just after different stimulations over the fifth time interval (the first time interval in the poststimulation period) on sustained attention, a two-tailed Wilcoxon signed-rank test on paired samples was conducted and the results showed that the median relative power change of the tACS group had no significant difference with that of the sham group, *p* = 1, corresponding to an effect size *r* = 0. These results indicated that tACS did not modulate power in pMFC when the tACS was just terminated (Figure 6(d)). On the other hand, Bayesian analysis showed very small evidence against the null hypothesis that sustained attention was modulated in tACS condition (BF = 0.31).

#### 3.2.3. Phase-Based Connectivity

A two-way repeated measures ANOVA was run to determine the effect of different stimulations (sham/tACS) over time intervals (20-25 min and 25-30 min) on the averaged dWPLI changes relative to the baseline (0-5 min) within the time-frequency window (150-300 ms, 5-8 Hz) determined in Experiment 1 (Figure 6(e)). The interaction effect between stimulation and time interval on averaged power was not statistically significant, *F* (1, 11) = 1.837, *p* = 0.203, partial *η*^2^ = 0.059. The main effect of stimulation was nonsignificant, *F* (1, 11) = 0.007, *p* = 0.924, partial *η*^2^ = 0.00013. The main effect of time was nonsignificant, *F* (1, 11) = 0.108, *p* = 0.749, partial *η*^2^ = 0.002. To specifically see the immediate effect just after different stimulations over the fifth time interval (the first time interval in the poststimulation period) on sustained attention, a right-tailed Wilcoxon signed-rank test on paired samples was conducted and the results showed that the relative dWPLI change of the sham condition was significantly larger than that of the tACS group, *p* = 0.026, corresponding to an effect size *r* = 0.566 (a medium effect). These results indicated that tACS reduced the phase-based connectivity between pMFC and LPFC when the tACS was just terminated (Figure 6(f)). A similar conclusion was reached by Bayesian analysis, which showed moderate evidence against the null hypothesis that phase-based connectivity was up(non)-regulated in tACS condition (BF = 5.48).

## 4. Discussion

To investigate pMFC-LPFC oscillations in the process of sustained attention, we first analyzed the correlation between theta characteristics (time-frequency power and phase-based connectivity) and the level of sustained attention and then utilized tACS to modulate theta characteristics and in turn observed its effects on sustained attention. In Experiment 1, two interested time-frequency windows were determined, in which high/low time-frequency power and high/low phase-based connectivity (indexed by dWPLI) corresponded to high/low-level sustained attention. In Experiment 2, time-frequency power and phase-based connectivity were compared between sham stimulation and tACS groups within the time-frequency window determined in Experiment 1. There was no significant difference in time-frequency power between the two stimulation groups. However, phase-based connectivity between pMFC and LPFC significantly decreased in the tACS group compared with the sham group during the first five minutes of the poststimulation period. Moreover, there was a marginal trend that sustained attention was downregulated by tACS in the same time interval, suggesting that theta phase synchronization between pMFC and LPFC may play a causal role in sustained attention.

In Experiment 1, the reaction time gradually increased as the experimental time went on, suggesting that the level of sustained attention gradually went down. This phenomenon, called vigilance decrement, was commonplace in PVT tasks [2]. Corresponding characteristics, including time-frequency power and phase-based connectivity, also showed consistency with previous studies. Frontal theta has been regarded as a crucial mechanism for cognitive control [35]. Ample studies suggested that external stimuli can evoke various event-related potentials, such as N2 and ERN (error-related negativity) components, which could reflect the process of cognitive control [27, 28]. A larger level of sustained attention evoked greater N2 amplitude and induced larger fm-theta power, representing a higher demand for cognitive control [35]. This mechanism could be well supported by the results of the time-frequency power shown in Experiment 1. In terms of phase-based connectivity, information was integrated in a short time to make decisions quickly in cognitive tasks. Research has shown that this process was mainly performed through phase synchronization between various brain areas [36]. The response to make as quickly as possible in PVT task involved the functional integration of many distributed areas, especially pMFC and LPFC. It had been shown that pMFC exerts control on attention by coordinating its activity with LPFC, which then conveys modulatory signals to low-level sensorimotor areas [37]. Higher synchronization may represent a higher level of control, as indicated by phase-based connectivity results in Experiment 1.

In Experiment 2, there were no significant differences in time-frequency power and performance of sustained attention between the sham and tACS groups. However, trends were shown that in the first five minutes during the poststimulation period, namely, 20-25 min (the fifth time interval), sustained attention was probably downregulated by tACS. Most importantly, in the fifth time interval, phase-based connectivity between pMFC and LPFC significantly decreased in the tACS group compared with the sham group. These facts probably implied the causal relationship between sustained attention and theta phase synchronization between pMFC and LPFC. A large number of studies suggested that tACS with different phase differences can manipulate phase synchronization [11, 29, 30]. For example, theta tACS with 0° phase difference increased frontotemporal synchronization and significantly improved working memory in older adults [12]. On the contrary, theta tACS with 180° phase difference desynchronized frontoparietal areas and caused decreased memory performance [38]. Given that tACS with 180° phase difference was utilized in Experiment 2, the significant difference across the two groups indicated that phase synchronization was also downregulated. As a result, we suspected that phase synchronization between pMFC and LPFC plays not only correlated but also causal roles in sustained attention. In terms of time-frequency power, our results showed that tACS did not have a modulation effect. Previous studies have shown that tACS can entrain oscillations, such as alpha oscillations [39, 40], but there are also inconsistent findings [41, 42]. On the other hand, the absence of time-frequency power in our study highlighted the exclusively causal relationship of phase synchronization in sustained attention.

There have been several similar studies in which theta band tACS over the pMFC was used to modulate sustained attention. For example, Rostami et al. aimed to modulate pMFC to influence sustained attention [13]. They found an increase in frontal theta power and alpha phase synchronization between central and parietal areas. Sustained attention was upregulated as well. The main difference between our study and Rostami et al.'s lied in the tACS electrode placements. We stimulated both pMFC and LPFC, thereby providing novel evidence for the phase synchronization between the two areas. Another study showed no modulation effect of sustained attention when 4 Hz tACS was exerted between electrodes FCz and Cz and two reference electrodes were placed on the cheeks [14]. We argued that the complexity showed by these studies including ours highlighted the importance of electrode placements, which implied distinct underlying mechanisms.

There are also some limitations to our study. The first limitation is our sample size across two experiments. We recruited 10 subjects in experiment 1 and 15 subjects (only 12 could be analyzed) in Experiment 2. It is better to collect more data to get more robust results, especially for signal analysis in tACS. The second limitation of our study is the lack of a 0° tACS comparison set in Experiment 2. tACS with 180° phase difference used in our study mainly came from the bipolar setting of the stimulator. Next, high-density tACS could be used to realize 0° tACS [12], providing more comprehensive evidence that theta phase synchronization plays a causal role in sustained attention. The third limitation is the lack of a control frequency. Similar to previous tACS studies [43–46], we compared stimulation effects between a frequency of interest and sham condition, without involving any control frequencies to rule out confounding effects brought by the frequency factor [47–48]. Future study could provide more convincing evidence of frequency-specific effects by introducing a control frequency condition.

## 5. Conclusions

The present study is aimed at investigating the causal roles of theta-band pMFC-LPFC oscillations in sustained attention via tACS. Results showed that in the first five minutes after tACS was terminated, theta-band phase-based connectivity between pMFC and LPFC significantly decreased; meanwhile, sustained attention had a declining trend. These findings implied the causal relationship between sustained attention and theta phase synchronization between pMFC and LPFC.

## Figures and Tables

**Figure 1:** Schematic illustration of one trial in Experiment 1.

**Figure 2:** Schematic illustration of Experiment 2: (a) timeline of experiment events; (b) schematic illustration of one trial.

**Figure 3:** The behavioral results in Experiment 1. (a) The averaged RTs were increasingly longer with the experimental time going on. Note the length of error bars is the standard deviation. (b) The averaged RTs of high-level sustained attention trials were significantly faster than those of low-level sustained attention trials (*t* (9) = −30.42, *p* < 0.0001).

**Figure 4:** Time-frequency power of pMFC (Fz). The power of (a) high-level and (b) low-level sustained attention (here abbreviated as SA) was computed by averaging across all subjects. (c) Districts circled in thin lines denote a significant difference between high-level and low-level sustained attention (high-level minus low-level). The bold black rectangle shows the interested time-frequency window (150-350 ms and 4-6 Hz). (d) The averaged power of high-level sustained attention was significantly larger than that of low-level sustained attention, *t* (9) = 3.30, *p* < 0.01.

**Figure 5:** Phase-based connectivity between pMFC (Fz) and LPFC (F3). DWPLI of (a) high-level and (b) low-level sustained attention (here abbreviated as SA) was computed by averaging across all subjects. (c) The difference between high-level and low-level sustained attention (high-level minus low-level) was demonstrated. The bold black rectangle shows the interested time-frequency window (150-300 ms and 5-8 Hz). (d) The averaged dWPLI of high-level sustained attention was significantly larger than that of low-level sustained attention, *t* (9) = 2.68, *p* < 0.05.

**Figure 6:** (a) Sustained attention in the two stimulation groups (sham/tACS) both declined with experimental time going on. There were no significant interaction or stimulation effects, but there was a significant main effect of time intervals, and the post hoc comparisons can be found in Table 1. (b) Sustained attention in the tACS group had a declining trend compared to the sham group in the fifth time interval (20-25 min) when the tACS was just terminated, *p* = 0.068. (c) There were no main effects or interactions between stimulation and time intervals in power in 20-25 min (TI5) and 25-30 min (TI6) after stimulation. (d) There were no significant differences in power between sham and true tACS groups in the fifth time interval (20-25 min) when the tACS was just terminated, *p* = 1. (e) There were no main effects or interactions between stimulation and time intervals in phase-based connectivity (indexed by dWPLI) in 20-25 min (TI5) and 25-30 min (TI6) after stimulation. (f) Phase-based connectivity in the tACS group significantly decreased compared with the sham group in the fifth time interval (20-25 min) when the tACS was just terminated, *p* = 0.026.

**Table 1:** Multiple comparisons of time intervals in behavioral results.

Group 1	Group 2	Statistic	Significance
TI 1 (0-5 min)	TI 2 (5-10 min)	-3.46	∗
TI 1 (0-5 min)	TI 3 (10-15 min)	-4.09	∗∗
TI 1 (0-5 min)	TI 4 (15-20 min)	-3.71	∗
TI 1 (0-5 min)	TI 5 (20-25 min)	-5.07	∗∗∗
TI 1 (0-5 min)	TI 6 (25-30 min)	-5.54	∗∗∗
TI 2 (5-10 min)	TI 3 (10-15 min)	-2.63	**ns**
TI 2 (5-10 min)	TI 4 (15-20 min)	-1.83	**ns**
TI 2 (5-10 min)	TI 5 (20-25 min)	-3.22	**ns**
TI 2 (5-10 min)	TI 6 (25-30 min)	-5.18	∗∗∗
TI 3 (10-15 min)	TI 4 (15-20 min)	0.331	**ns**
TI 3 (10-15 min)	TI 5 (20-25 min)	-0.92	**ns**
TI 3 (10-15 min)	TI 6 (25-30 min)	-3.14	**ns**
TI 4 (15-20 min)	TI 5 (20-25 min)	-1.71	**ns**
TI 4 (15-20 min)	TI 6 (25-30 min)	-3.86	∗
TI 5 (20-25 min)	TI 6 (25-30 min)	-2.98	**ns**

Note: significant effects are marked by asterisks and bold text. ^∗∗∗^*p* < 0.001, ^∗∗^*p* < 0.01, and ^∗^*p* < 0.05. *p* values are Bonferroni corrected. TI denotes the time interval, e.g., TI 1 denotes the first time interval: 0-5 min.

## Data Availability

The data used to support the findings of this study are available from the corresponding author upon request.
